The article "Podophyllotoxin and Rutin Modulate M1 (iNOS+) Macrophages and Mitigate Lethal Radiation (LR) Induced Inflammatory Responses in Mice" was retracted in 2022. Reasons: concerns about the data; concerns about the images.

# Podophyllotoxin and Rutin Modulate M1 (iNOS+) Macrophages and Mitigate Lethal Radiation (LR) Induced Inflammatory Responses in Mice

**DOI:** 10.3389/fimmu.2019.00106

**Published:** 2019-02-12

**Authors:** Vinod Nadella, Rajiv Ranjan, Balasubramanian Senthilkumaran, S. S. Y. H. Qadri, Suresh Pothani, Ajay Kumar Singh, Manju L. Gupta, Hridayesh Prakash

**Affiliations:** ^1^Laboratory of Translational Medicine, School of Life Science, University of Hyderabad, Hyderabad, India; ^2^Institute of Nuclear Medicine and Allied Sciences, Defence Research and Development Organization, New Delhi, India; ^3^Department of Animal Biology, School of Life Sciences, University of Hyderabad, Hyderabad, India; ^4^National Institute of Nutrition, Indian Council of Medical Research Hyderabad, Hyderabad, India; ^5^National Animal Resource Facility for Bio-Medical Research, Indian Council of Medical Research Hyderabad, Hyderabad, India

**Keywords:** radiation syndrome, macrophages polarization, Th1/2 response, immune tolerance, radioprotection

## Abstract

Accidental exposure to lethal doses of Gamma radiation leads to the systemic inflammatory syndrome which causes mortality. In view of this, management of hemopoietic syndrome by modulating pro-inflammatory response in clinically manageable time period seems to be the most appropriate strategy for encountering radiation induced damage and recovery. As both tissue and peripheral macrophages are critical for the management of radiation induced injuries, we have unraveled the immunomodulatory potential of radioprotective formulation (G-003M) on peripheral macrophages populations in this study. G-003M inhibited lethal radiation induced NO and Th1 effector cytokines in the exposed macrophages indicating its M1 dim polarizing capacity. In similar lines, conditioning of mice with G-003M before lethal irradiation (LR) inhibited LR induced titre of Th1 effector cytokines in both serums as well as in lung, small intestine, and spleen tissue confirming its immunomodulatory potential. G-003M potentially down modulated inflammatory response in LPS induced inflammatory model and enhanced M2 polarization of iNOS+ M1 effector macrophages providing a molecular hint on G-003M mechanism of action on macrophages. These observations revealed that G-003M potentially modulate pro-inflammatory programming of macrophages and mitigate radiation-induced inflammatory stress which is believed to contribute significantly to radioprotective attribute of G-003M. In this study, we demonstrate that Rutin and Podophyllotoxin drive M1^dim^/M2 polarization of LR primed macrophages apart from protecting DNA from radiation. These drugs have the capacity to programme innate immune cells like macrophages which may be involved in homeostasis during recovery.

## Introduction

Immunosuppression, opportunistic infections and deleterious inflammation are the most important manifestations of exposure to high doses of low LET radiations (1). These leads to hemopoietic and gastrointestinal syndrome which ultimately leads to the death of exposed individuals (2, 3). Out of these, hemopoietic syndrome is fairly repairable if managed within an amicable post irradiation time, thus offering therapeutic benefits. Various immunomodulators including Glucan, Amifostin, WR2721, LPS, and Interleukin-1 have been explored as radioprotectors which enhanced survival by enhancing the hemopoietic recovery (4–8) by their capacity to enhance secretion of various cytokines which can stimulate monocytes / macrophages (9, 10).

We have recently demonstrated the radioprotective potential of Podophyllotoxin and Rutin formulation (G-003M) which was prepared from radioprotective plant e.g., *Podophyllum hexandrum* (11–18) in mice model system (19). G-003M is known to protect mice from respiratory syndrome and fibrosis by down regulating inflammatory response in mice (20). On these bases, we anticipated that these formulations may reduce inflammatory response in the macrophages which may account for their radioprotective mechanism. Therefore, we analyzed immunomodulatory role of G-003M on macrophages populations which are sentinels of inflammatory responses (21) and important for tissue homeostasis, host defense against tissue insult and infections (22–24).

Macrophages based therapeutic interventions for the management of various diseases have gained significant attention in recent years (25). This is mainly attributed to high degree of plasticity and functions which are collectively required for radioprotection (26, 27). Both phenotypical and functional plasticity of macrophages (28–30) enable them to perform wide range of functions which are required for protecting tissue from radiation damage. Both M1 and M2 types of macrophages differ in the expression of iNOS proteins which are key characteristic of M1 effector macrophages. Resting and iNOS^−^macrophages get activated and become iNOS^+^ macrophages which are also known as M1 effector (27, 29, 31) and drive Th1 inflammatory response post irradiation and expected to contribute to radiation induced inflammatory syndrome. In contrast, M2 macrophages are alternatively activated macrophages and drive Th2 immune responses which are predominately anti-inflammatory and regenerative in nature and anticipated to contribute to radio recovery. From this point of view, we expected possible modulation of M1 effector phenotype of macrophage by G-003M in irradiated mice. Following our expectation, G-003M mitigated lethal radiation induced NO and secretion of Th1 effector cytokines in the cell culture supernatants of irradiated CD11b+ primary macrophages. Similarly, pre-irradiation conditioning of mice with G-003M inhibited LR induced Th1 cytokines in both serum as well various vital tissues analyzed thus proved immunomodulatory potential of G-003M. Apart from the lethal radiation, G-003M retuned M1 effector macrophages in LPS treated/challenged mice model as well providing the molecular hint on underlying immunological mechanism which need further investigation.

Taken together these observations revealed G-003M driven inflammatory programming of lethally irradiated macrophages during radiation-induced inflammatory response and believe that this may contribute significantly to radioprotective attribute of G-003M.

## Results

### Rutin and Podophyllotoxin Promote M2 Polarization of Th1 Primed Macrophages

Any radioprotective formulation should not only protect DNA from damage but also changes the redox status of cells and bring down the inflammatory response. With this mandate, we argued whether Podophyllotoxin and Rutin, apart from being anti-oxidant and radioprotective in nature, would also harbor anti-inflammatory potential or not. In order to demonstrate the immune mediated mechanism of radioprotective formulations viz Rutin, Podophyllotoxin; we investigated the impact of these formulations on macrophages which are important for radioprotection. Podoglucoside being one of the active compounds of Podophyllum hexandrum, along with Rutin and Podophyllotoxin, we included Podoglucoside to our experiment as control while analysing the impact of these compounds individually. Treatment of macrophages with Rutin, Podophyllotoxin, and Podoglucoside inhibited the generation of NO (an indicator parameter of macrophage activation) in the cell culture supernatants of naïve macrophages and more strongly in Th1 primed macrophages (Figures 1A–D and Supplementary Figures 1A–D) suggesting M1 dim or M2 polarizing capacity of these formulations in M1macrophages. To further confirm the impact of these formulations on M1/M2 polarization, we analyzed various M1/M2 effectors proteins in these macrophages. These formulations, in line with NO, also inhibited the expression of iNOS (M1 effector protein) and other key signaling proteins including pp38 MAPK, phospho STAT3 and phospho NF-kB (Figure 1 and Supplementary Figure 1) which are critical for the translational of iNOS protein and M1 effector immune response in inflammatory macrophages. To further confirm the impact of these formulations *in vivo* we analyzed their impact on primary macrophages as well which actually sense radiation stress during exposure. To this end, we harvested and purified CD11b+ peripheral macrophage by CD11b+ microbeads (Miltenyi Biotech). These macrophages were stimulated with LPS, IFNγ, and/or LPS+IFNγ and subsequently treated with formulations. Interestingly, and in line with RAW macrophages, these formulations consistently inhibited the generation of NO in their cell culture supernatant as well as the expression of key signaling proteins including phospho p38 MAPK, pSTAT3, and NF-kB (Figure 2 and Supplementary Figure 2) thus confirmed their immunomodulatory role on M1 response *in vivo* as well. Furthermore, our data revealed that these formulations also upregulated the expression of CD206 and Arginase (M2 effector proteins) in both RAW and CD11b+ primary macrophages providing the evidence of M2 polarizing / scavenging capacity of Rutin and podophyllotoxinin macrophages which was in accordance of our original hypothesis.

**Figure 1:** Rutin and Podophyllotoxin promote M2 polarization of Th1 primed RAW264.7 macrophages. RAW macrophage cell line (RAW 264.7) were stimulated without **(A)** and with pro-inflammatory cytokines including LPS **(B)**, IFNγ **(C)**, and LPS+IFNγ **(D)** and were treated with formulations for 24 h. Cell culture supernatants were collected and analyzed for nitrite/nitrate as a surrogate marker of NO. Shown here is the mean μM of NO ± S.E. from 3 independent replicates. Whole cell lysates from these cells were prepared and various signaling and M1 effector proteins were analyzed by western blotting. β-actin was used as a loading control. Shown here is the representative of 4 independent experiments with similar outcome. The Western blots were quantified for densitometry by Image J software, and mean densitometry values of independent proteins was normalized with the mean densitometry values of its respective β-actin band intensity value to present the relative expression of each protein as a mean in the ratio of protein to actin. Statistical analysis was conducted using ANOVA followed by Dunnett's post-test (^*^p ≤ 0.05, ^**^p ≤ 0.01, ^***^p ≤ 0.001).

**Figure 2:** Rutin and Podophyllotoxin promote M2 polarization of Th1 primed CD11b+ primary macrophages. CD11b+ peritoneal macrophages from C57BL/6J mice were stimulated without **(A)** and with pro-inflammatory cytokines including LPS **(B)**, IFNγ **(C)** and LPS+IFNγ **(D)** and were treated with formulations for 48 h. Cell culture supernatants were collected and analyzed for nitrite/nitrate as a surrogate marker of NO. Shown here is the mean μM of NO ± S.E. from 3 independent replicates. Whole cell lysates from these cells were prepared and various signaling and M1 effector proteins were analyzed by western blotting. β-actin was used as a loading control. Shown here is the representative of 4 independent experiments with similar outcome. The Western blots were quantified for densitometry by Image J software, and mean densitometry values of independent proteins was normalized with the mean densitometry values of its respective β-actin band intensity value to present the relative expression of each protein as a mean in the ratio of protein to actin. Statistical analysis was conducted using ANOVA followed by Dunnett's post-test (^*^p ≤ 0.05, ^**^p ≤ 0.01, ^***^p ≤ 0.001).

### Rutin Promotes M2 Polarization of Peripheral Macrophages During Systemic Inflammatory Response

Radiation is a non-specific stimulus and triggers multiple events for the response. To explore the probable and specific mechanism by which these drugs can modulate macrophages phenotype, we used LPS induced systemic inflammation (32) model in mice. To this purpose, C57Bl/6j mice were treated with LPS (10 mg/KBW) in presence of Rutin and peripheral macrophage infiltration as well as their polarization was analyzed as depicted in Figure 3A. FACS analysis revealed that exposure of mice to LPS increased peripheral infiltration of CD11b+ macrophages from day 1 through day 7 post treatment as an index of systemic pro-inflammatory response in these mice (Figure 3B). Although conditioning of these mice with Rutin enhanced peripheral infiltration of CD11b+ macrophages from day 1 through day 3 post treatments, but got reduced by day 7 post treatment indicating immunomodulatory potential of Rutin in these inflamed mice (Figure 3B). On these bases, we anticipated similar response in T cell populations in the peritoneal lavage. However, and to our surprise, the number of CD4+ and CD8a+ single T cells populations remained unchanged in these mice during the course of experiments. Although there is a steady increase in CD4 population by Rutin in LPS treated mice (Supplementary Figures 3A–C) in comparison to placebo, but that remained insignificant and during the course of experiment in these mice. We further analyzed the purified CD11b+ macrophages from these mice and found a clear inhibition of LPS induced expression of iNOS (M1) and associated signaling proteins and concomitant upregulation of Arginase and CD206 (M2 effector proteins) by Rutin (Figure 3C). These results potentially demonstrated immunomodulatory potential of Rutin in skewing refractory and scavenging phenotype in macrophages which are potentially homeostatic in nature and could contribute to the radioprotection.

**Figure 3:** Rutin modulate innate as well adaptive immunity during systemic inflammation. **(A)** C57BL/6J mice were treated with LPS (1 μg/ml) in the presence and absence of Rutin. Mice were euthanized for peritoneal lavage on day 1st, 3rd, and 7th post irradiation; Schematic representation. **(B)** Peritoneal lavage was analyzed by FACS for CD11b+ macrophages, and percentage positive cells were plotted. **(C)** CD11b+peripheral macrophages from mice day 7 post treatments were lysed and analyzed for various signaling, M1, and M2 effector proteins by Western blotting. β-actin was used as a loading control. Shown here is the representative of 3 independent experiments with similar outcome. The Western blots were quantified for densitometry by Image J software, and mean densitometry values of independent proteins were normalized to its mean densitometry values of its respective β-actin band intensity value to present the relative expression of each protein as a mean in the ratio of protein to actin. Statistical analysis was conducted using ANOVA followed by Dunnett's post-test (^**^p ≤ 0.01, ^***^p ≤ 0.001).

### G-003M Modify Immune Response of Lethally Irradiated Macrophages

On the basis of M2 polarizing capacity of Rutin and Podophyllotoxin, we anticipated that these formulations would modulate gamma irradiation induced inflammatory responses as well. To that purpose, the impact of these formulations on gamma irradiated CD11b+ primary macrophages was analyzed as per Figure 4A. Thioglycolate elicited macrophages from C57Bl/6j mice were purified by CD11b MACS beads and subsequently cultured, stimulated withTh1 priming conditions as explained elsewhere. These cells were subsequently treated with either G-003M or Quercetin (as a positive control), 1 h before irradiating them with LR dose using 60 Cobalt gamma chamber, Cobalt teletherapy, Bhabhatron II. In line with our hypothesis and previous data, both G-003M and/or Quercetin inhibited LR/LPS/IFNγ induced NO titres in the culture supernatant of these macrophages at various time intervals (Figure 4B) indicating the M1^dim^ phenotype of drug pulsed macrophages. Further analysis of Th1 effectors cytokines revealed anti-inflammatory impact of G-003M and/or Quercetin in Th1 primed or LR irradiated macrophages (Figures 5A–C). Out of various cytokines we analyzed, inhibition of IFNγ by G-003M (Figure 5B) particularly confirmed anti-inflammatory and cytoprotective action of G-003M which corroborated *in vitro* findings *in vivo*.

**Figure 4:** G-003M inhibit macrophages activation during gamma irradiation. **(A)** Peripheral CD11b+ macrophages were harvested fromC57BL/6Jmice using thioglycolate based method and cells were treated with G-003M 1 h before irradiated with 9Gy dose. These cells were then stimulated with pro-inflammatory cytokines and cultured for indicated time intervals; Schematic representation. **(B)** Cell culture supernatants were collected at indicated time intervals and analyzed for nitrite/nitrate as a surrogate marker of NO. Shown here is the mean μM of NO and/or pg of cytokines produced ± S.E. from 3 independent replicates. Statistical analysis was conducted using ANOVA followed by Dunnett's post-test (^*^p ≤ 0.05, ^**^p ≤ 0.01, ^***^p ≤ 0.001).

**Figure 5:** G-003M inhibit Th1 effector response in lethally irradiated macrophages. Cell culture supernatants from macrophages used in Figure 4 were collected at indicated time intervals and various Th1 effector cytokines including **(A)** TNFα **(B)** IFNγ and **(C)** Il-6 were analyzed by standard ELISA method. Shown here is the mean or pg of cytokines produced ± S.E. from 3 independent replicates. Statistical analysis was conducted using ANOVA followed by Dunnett's post-test (^*^p ≤ 0.05, ^**^p ≤ 0.01, ^***^p ≤ 0.001).

### G-003M Potentially Down Modulate Inflammatory Response of Lethally Irradiated Animals

Observed anti-inflammatory potential of G-003M in purified macrophage populations provoked us to test the same *in vivo*. For that purpose, mice were conditioned with G-003M, 1 h before irradiating them with LR using 60 Cobalt gamma chamber, Cobalt teletherapy, Bhabhatron II. Mice were euthanized and critical organs like lungs, intestine and spleen which are sensitive for radiation damage were analyzed for inflammatory response as per scheme shown in Figure 6A. Systemic irradiation of mice with LR enhanced the pulmonary levels of both TNF-α (Figure 6B) and IFNγ (Figure 6C) indicating pulmonary fibrosis in these mice as cellular damage upon irradiation is known to result in cytokine-mediated induction and progression of inflammatory and fibrotic tissue reactions (33, 34). In line with our *in vitro* data and in accordance of our hypothesis, G-003M inhibited the titre of these Th1 cytokines in the lungs. Splenic tissue however remained redundant for G-003M driven changes in these cytokines which could be due to sterile nature of spleen. Systemic increase of IFNγ in context of radiation exposure contributes to the radio sensitization of small intestine tissue in particular. Interestingly, G-003M mediated drop in IFNγ titres in all three organs tested (Figure 6C) potentially indicates its anti-inflammatory action contributing to radioprotection.

**Figure 6:** G-003M potentially inhibit inflammatory response of lethally irradiated animals. **(A)** C57BL/6J mice were injected G-003M intramuscularly 1 h before irradiated with 9Gy dose. Mice were euthanized at indicated time intervals for lung, spleen, and small intestine; Schematic representation. Tissue lysates were analyzed for various pro-inflammatory cytokines including **(B)**TNF-α, **(C)** IFNγ, and **(D)** IL-6 in lung, small intestine and spleen by ELISA. **(E)** Serum titres of TNF-α, IFNγ, and IL-6 were also quantified in serum samples of the same mice by ELISA. Shown here is the mean pg of cytokines produced ± S.E. from 3 independent replicates. Statistical analysis was conducted using ANOVA followed by Dunnett's post-test (^*^p ≤ 0.05, ^**^p ≤ 0.01, ^***^p ≤ 0.001).

To further substantiate, titres of IL-6, a double edge cytokine which promote both Th1 in normal and Th2/17 response in damaged organs thus contributing to tissue fibrosis during lethal radiation was analyzed. Systemic irradiation of mice with LR enhanced the secretion of IL-6 transiently in both lung and intestine (Figure 6D). Interestingly and in line with G-003M effect on IFNγ and TNF-α titres, G-003M inhibited IL-6 titres particularly in small intestine of lethally irradiated mice. Furthermore, significant inhibition in serum values of these Th1 effector cytokines particularly TNF-α and IFNγ by G-003M formulations in lethally irradiated mice (Figure 6E) provided a compelling evidence of anti-inflammatory manifestation of G-003M in lethally irradiated mice and corroborated our *ex vivo* findings on peritoneal macrophages. On the basis of these results, we strongly anticipate that this formulation, other than protecting DNA from radiation induced damage, would also promote the polarization of M1 macrophages toward M2 phenotype which may add to the mechanisms of radioprotection. This is quite relevant hypothesis which may account most for underlying mechanism of protection of these tissues by G-003M thus warrant further study.

## Discussion

Radiation induced syndromes are manifested by the inflammatory responses which are damaging and destructive in nature. Therefore, modulating Th1 inflammatory response is one of paramount requirement for the radioprotection and subsequent recovery. Macrophages based therapeutic interventions for various diseases models have gained significant attention in recent years since these are capable of orchestrating the immune response as seen in many disease models (25). In contrast to dendritic cells (DCs), macrophages display a range of phenotypic plasticity (M0, M1, M2a 2b, 2c) with an entire range of physiological and immunological functions (26, 27) which may afford protection from radiation damage.

Unlike gastric or central nervous syndrome, hemopoietic syndrome is repairable within an amicable post irradiation time. We strongly believe that selective retuning of M1 effector macrophages to M2 post radiation exposure would not only be effective in managing hemopoietic but also gastric syndrome as well for recovery. This is due to strong anti-inflammatory and angiogenic nature of M2 macrophages which are anticipated to promote recovery of GI track particularly intestinal villi by activating paneth cell proliferation. We have previously demonstrated that radioprotective potential of G-003M to mice was by efficient scavenging of ROS, regulating various pro-apoptotic and anti-apoptotic proteins. However, we also believe that those protective mechanisms may not be just sufficient for protecting the tissue from radiation damage and we argued that its radioprotective mode of action may also include *in situ* programming of macrophages which are fairly radio resistant and available for the intervention during sequel of damage (32, 35, 36).

G-003M driven reduced infiltration of CD11b+ macrophages in LPS challenged mice not only confirmed its anti-inflammatory role but also provided a probable immune mechanism. LPS is known to bind CD14+ macrophages and trigger TLR2/4 mediated immune response during Th1 inflammatory response in the gut. The infiltrating macrophages induce the expression of iNOS and become regulatory to various pathogens which often infiltrate out of gut during radiation syndrome. In order to overcome radiation induced gastritis, anti-inflammatory drugs have been explored like DMRD and/or Immune complex. In this context, G-003M driven expression of M2 phenotype markers including Arginase and CD206 potentially demonstrated that G-003M programmed M2 macrophages would not only down regulate inflammatory response but also potentially remove cellular debris and help in homeostasis. In line with LPS response on macrophages, irradiation of primary macrophages or macrophages from irradiated mice induced iNOS and downregulated the expression of molecules that convey an M2 phenotype, including CD206 and Arginase. Thus, these results potentially indicated that Rutin can be used for various palliative therapies as well for other inflammatory conditions/pathologies. G-003M driven M2 polarization of Th1/LR exposed M1 macrophages also provided a possible hints of its action on TLR 2/4 mediated signaling pathways which was evident by reduced expression of signaling proteins in Th1 effector macrophages (37).

G-003M mediated drop of IFNγ and IL-6 response, and concomitant upregulation of CD206 furthermore demonstrated that G-003M can potentially transform these inflammatory macrophages into scavenging macrophages which are important for tissue homeostasis in the irradiated tissue microenvironment. Therefore, we strongly believe that increased infiltration of CD169+ macrophages in G-003M treated animals contribute to tissue protection. On the basis, it is evident that G-003M, other than protecting DNA from radiation induced damage, also contributes to inflammatory programming of macrophages for reconstitution of damaged organs in the course of radioprotection. Moreover, we also anticipate G-003M mediated differentiation of effector T cells toward regulatory T cells as our recent study suggested that M1/M2 macrophage have the ability to support Th1/Th2 responses.

From this work, it is quite evident that macrophages-based strategies would hold therapeutic potential in the management of radiation injuries and we anticipate that adoptive transfer of M2 macrophage in particular be one of the treatment modalities not only against planned but also unplanned exposure to radiations. This is very intriguing aspect of the study and warrant in depth analysis in future.

## Materials and Methods

### Antibodies and Reagents

The general reagents were purchased from Sigma-Aldrich (UK), unless stated otherwise. RPMI 1640, Lipopolysaccharide (LPS), Penicillin Streptomycin solution were procured from the Sigma-Aldrich. Recombinant mouse IFN cytokine is from eBiosciences, (San Diego, CA). CD11b+ human and Mouse MACS Microbeads and LC Columns are from MiltenyiBiotec. Primary antibodies including rabbit polyclonal NOS-2, rabbit polyclonal CD-206, rabbit polyclonal β-Actin, mouse monoclonal β-Actin are from Santa Cruz biotechnology. Mouse monoclonal Arginase-1 is from BD Biosciences. Rabbit monoclonal pSTAT3, p38MAPK, and pNF-kB p65 are from Cell Signaling Technology. HRP-linked anti-mouse IgG and anti-rabbit IgG are from Cell Signaling Technology. Anti-mouse/human-CD11b (Clone (M1/70)-FITC-conjugated, anti-mouse CD4 (Clone GK1.5)-PE-conjugated, and anti-mouse-CD8a (Clone 53-6.7)-Per CP/cy5.5-conjugated antibodies and their respective isotype control anti-body including FITC Rabbit IgG2bK (Clone RTK4530), PE Rat IgG2bK (Clone RTH4530) and PerCP/Cy5.5 Rat IgG2bK (RTK4530) were procured from Biolegend (Germany). TNFα, IFNγ, and IL-6 ELISA kits were purchased from R&D system (Darmstadt, Germany).

### Preparation of Drug Formulations and G-003M Formulation

Podophyllotoxin and Rutin at 1:2 ratio (G-003M) was prepared by dissolving both the compounds in PEG300. The solution was further diluted in distilled water to a final ratio of 1:9 (PEG300:water). The preparation was administered intramuscularly (150 μl per mice at a dose of 6.5 mg/kg body weight) 1 h prior to radiation exposure. The effective concentration of the formulation was obtained from the whole-body survival study (19). G-003M was freshly prepared every time and just before the time of administration.

### Animal Studies

All animal experiments were performed as per the guidelines laid down by institutional Animal ethical committee and approved by Institutional Animal ethical committee approval (**UH/IAEC/HP/2014-I/22**) to HPF or *in vivo* studies, C57/Bl6 mice were purchased from NIN, Hyderabad, were maintained at 20–22°C and relative humidity of 50–70%. Mice were given a standard diet of rodent pellets and water. Six to eight-week-old mice were kept in well-ventilated perplex boxes. Mice were sacrificed by cervical dislocation. CD11b+ macrophages were collected from mice peritoneal lavage and purified by MACS based method (Miltenyi Biotech) for analyzing various signaling proteins by western analysis. For radiation-based experiments, mice were randomly divided into four groups (Sham, G-003M only, 9Gy only and G-003M + 9Gy) with six mice in each group and exposed the radiation only groups to whole-body gamma irradiation (9Gy) in the Co-60 Cobalt gamma chambers (Cobalt Teletherapy, Bhabhatron II, Panacea Medical Technologies Pvt. Ltd., India) at a dose rate of 1.038 Gy/min. The exposure window and source to surface distance was 35 × 35 and 120 cm, respectively. Immediately after irradiation, mice were returned to the cage and rested. Radiation dose calibration was performed by the institutional radiation physicists at regular time intervals by Frick's dosimetry. Animals were sacrificed on day 1, day 3, and day 7 for peritoneal lavage, serum, lung, spleen, and small intestine.

### Primary Cell Isolation and Purification

To isolate CD11b+ peritoneal macrophages, C57BL/6J mice were injected with 1 ml of 4% brewer thioglycolate medium intra peritoneally and peritoneal lavage was harvested at third day post injection. Peritoneal lavage was centrifuged at 1,500 rpm for 8 min and the cells pellet was resuspended in fresh serum free RPMI. CD11b+ macrophages were purified by MACS-based separation method and were cultured in serum containing medium overnight. Macrophage monolayers were washed on the following day once with serum-free medium to remove any unbound cells. Cells were stimulated with LPS, IFNγ or both with or without formulations and cultured for 24 h. In radiation-based experiments cells were treated with formulation 1 h prior to irradiation using Co-60 cells.

### Cell Culture

Standard murine macrophage cell line RAW264.7A, procured from ATCC, were cultured in RPMI-1640 medium containing 2 mM L-glutamine supplemented with 10% FCS, 100 IU/ml penicillin, and 100 μg/ml streptomycin. Mouse peripheral CD11b+ macrophages purified by MACS bead-based method (Miltenyi Biotech) were cultured at 37°C in a humidified environment at 5% CO_2_. Cells were seeded at 2.5 × 10^4^ cells per well in a 96 well plate and incubated o/n for adhesion. Cells were stimulated with either LPS (1 μg/ml), IFNγ (50 ng/ml) or both (LPS + IFNγ) with or without formulations at 100 ng/ml and cultured for 24 h, while un-stimulated cells were maintained as controls.

### Quantification of NO

Nitric oxide production in macrophage culture supernatants was quantified by standard Griess reagent method as nitrate Equal volumes of the culture supernatants and Griess reagent (1% sulphanilamide/0.1% N-(naphthyl) ethylene-diaminedihydrochloride prepared in 5% o-phosphoric acid) were mixed and incubated. Absorbance was recorded at 550 nm by TECAN multimode spectrophotometer. Nitrate titres as surrogate markers of nitric oxide production in samples were quantified against a NaNO_2_ standard curve generated using software provided with the TECAN multimode spectrophotometer.

### Western Analysis

RAW macrophage cell or CD11b+ primary macrophages from mice were lysed in RIPA buffer (50 mMTris–HCl, pH 7.4, 150 mM NaCl, 2 mM EDTA, 1% Nonidet P-40 and protease inhibitor mixture) and sonicated. The lysate was centrifuged at 14,000 rpm for 20 min at 4°C to separate the particulate fraction. Protein in cell lysates was quantified by the Bradford assay using multimode plate reader (TECAN). Cell lysates containing 25 μg of protein were dissolved with an equal volume of 2 × Laemmli buffer (Sigma), heated to 95°C for 5 min and resolved by standard SDS-polyacrylamide gel electrophoresis (Bio-Rad) and blotted on PVDF membranes. Blots were blocked at room temperature for 1 h with 5% non-fat dry milk in TBS-T (20 mM Tris base, 137 mM NaCl and 0.05% Tween 20, pH 7.5) and incubated overnight at 4°C with primary and subsequently with horseradish peroxidase-conjugated secondary antibodies. Blots were developed by using ECL (Millipore) reagent and normalized against β-actin.

### Cytokine Quantification

Cytokines were quantified using sandwich ELISA kit (R&D system, Darmstadt, Germany) as per the instruction manual from manufacturer.

### Flow Cytometric Analysis

For the fluorescence-activated cell sorting (FACS) analysis, 1 × 106 viable peritoneal macrophages were washed with the ice-cold phosphate buffer and fixed in 70% ethanol. Cells were then blocked with FACS buffer (2% fecal calf serum in PBS) for 30 min. After blocking, cells were stained with FITC anti-mouse CD11b (Clone M1/70), PE anti-mouse CD4 (Clone GK 1.5) and PerCp/Cy5.5 anti-mouse CD8a for 20 min on ice in FACS buffer. Cells were washed in ice cold PBS twice and were analyzed using FACS ARIA II (BD Pharmingen). FACS data were analyzed by FlowJo software V10.

### Statistical Analysis

All results were expressed as the mean ± SEM of several independent experiments performed. Statistical analysis was conducted using two-tailed unpaired *t-*test for two data sets and 2-way ANOVA followed by Bonferroni post-test was used for multiple group comparisons (^*^P < 0.05; ^**^P < 0.01; ^***^P < 0.001). All the statistical analysis was carried out with GraphPad Prism Version 5.0 software.

## Author Contributions

VN conducted the experiments, analyzed the data, and designed the figures. RR provided technical assistance in radiation-based experiments. BS, SQ, SP, AS, and MG contributed reagents, materials, and analysis tool. HP conceived the idea. VN and HP wrote the paper.

### Conflict of Interest Statement

The authors declare that the research was conducted in the absence of any commercial or financial relationships that could be construed as a potential conflict of interest. The reviewers AG, MP and handling editor declared their shared affiliation.

## Supplementary Material

Supplementary Figure 1 Rutin and Podophyllotoxin promote M2 polarization of Th1 primed macrophages. RAW macrophage cell line (RAW 264.7) were stimulated without **(A)** and with pro-inflammatory cytokines including LPS **(B)**, IFNγ **(C)**, and LPS_IFNγ **(D)** and were treated with formulations for 48 h. Cell culture supernatants were collected and analyzed for nitrite/nitrate as a surrogate marker of NO. Shown here is the mean μM of NO ± S.E. from 3 independent replicates. Whole cell lysates from these cells were prepared and various signaling and M1 effector proteins were analyzed by western blotting. β-actin was used as a loading control. Shown here is the representative of 4 independent experiments with similar outcome. The Western blots were quantified for densitometry by Image J software, and mean densitometry values of independent proteins were divided with its mean densitometry values of its respective β-actin band intensity value to present the relative expression of each protein as a mean in the ratio of protein to actin. Statistical analysis was conducted using ANOVA followed by Dunnett's post-test (^*^*p* ≤ 0.05, ^**^*p* ≤ 0.01, ^***^*p* ≤ 0.001).

Supplementary Figure 2 Rutin and Podophyllotoxin inhibit Th1 primed CD11b+ primary macrophages. RAW macrophage cell line (RAW 264.7) were stimulated without **(A)** and with pro-inflammatory cytokines including LPS **(B)**, IFNγ **(C)**, and LPS_IFNγ **(D)** and were treated with formulations for 24 h. Cell culture supernatants were collected and analyzed for nitrite/nitrate as a surrogate marker of NO. Shown here is the mean μM of NO ± S.E. from 3 independent replicates. Statistical analysis was conducted using ANOVA followed by Dunnett's post-test (^*^*p* ≤ 0.05, ^**^*p* ≤ 0.01, ^***^*p* ≤ 0.001).

Supplementary Figure 3 Rutin potentially enhances peripheral CD11b+ population in mice treated with LPS. C57BL/6J mice were treated with LPS (1 g/ml) in the presence and absence of Rutin. Peritoneal lavage collected from these mice on day 1 **(A)**, day 3 **(B)**, and Day 7 **(C)** were analyzed by FACS for CD11b+ macrophages, CD4 and CD8a population. Percentage CD4 and CD8a positive cells were plotted. Shown here the representative FACS plots from each experimental group.

## References

[1] GrossmanSAYeXLesserGSloanACarrawayHDesideriS. Immunosuppression in patients with high-grade gliomas treated with radiation and temozolomide. Clin Cancer Res. (2011) 17:5473–5480. 10.1158/1078-0432.CCR-11-077421737504PMC3156964

[2] TravisELPetersLJMcNeillJThamesHDKarolisC. Effect of dose-rate on total body irradiation: lethality and pathologic findings. Radiother Oncol. (1985) 4:341–51. 10.1016/S0167-8140(85)80122-53909241

[3] GottlöberPSteinertMWeissMBebeshkoVBelyiDNadejinaN. The outcome of local radiation injuries: 14 years of follow-up after the Chernobyl accident. Radiat Res. (2001) 155:409–16. 10.1667/0033-7587(2001)155[0409:TOOLRI]2.0.CO;211182791

[4] Vijay-KumarMAitkenJDSandersCJFriasASloaneVMXuJ. Flagellin treatment protects against chemicals, bacteria, viruses, and radiation. J Immunol. (2008) 180:8280–5. 10.4049/jimmunol.180.12.828018523294

[5] NetaRWilliamsDSelzerFAbramsJ. Inhibition of c-kit ligand/steel factor by antibodies reduces survival of lethally irradiated mice. Blood (1993) 81:324–7. 7678509

[6] NetaROppenheimJJSchreiberRDChizzoniteRLedneyGDMacVittieTJ. Role of cytokines (interleukin 1, tumor necrosis factor, and transforming growth factor beta) in natural and lipopolysaccharide-enhanced radioresistance. J Exp Med. (1991) 173:1177–82. 10.1084/jem.173.5.11772022925PMC2118844

[7] KumagaiKIzumiHTsurusawaMMoriKJ. Radioprotection of LPS-resistant C3H/HeJ mice by RES-blockade. Experientia (1982) 38:861. 10.1007/BF019723187049723

[8] Lacave-LapalunJVBenderitterMLinardC. Flagellin and LPS each restores rat lymphocyte populations after colorectal irradiation. J Leukoc Biol. (2014) 95:931–40. 10.1189/jlb.041320924532644

[9] Lacave-LapalunJVBenderitterMLinardC. Flagellin or lipopolysaccharide treatment modified macrophage populations after colorectal radiation of rats. J Pharmacol Exp Ther. (2013) 346:75–85. 10.1124/jpet.113.20404023596059

[10] TakagiYChoiISYamashitaTNakamuraTSuzukiIHasegawaT. Immune activation and radioprotection by propolis. Am J Chin Med. (2005) 33:231–40. 10.1142/S0192415X0500288615974482

[11] KumarRSinghPKSharmaAPrasadJSagarRSinghS. *Podophyllum hexandrum* (Himalayan mayapple) extract provides radioprotection by modulating the expression of proteins associated with apoptosis. Biotechnol Appl Biochem. (2005) 42(Pt 1):81–92. 10.1042/BA2004016415762843

[12] DuttaAVermaSSankhwarSFloraSJGuptaML. Bioavailability, antioxidant and non toxic properties of a radioprotective formulation prepared from isolated compounds of Podophyllum hexandrum: a study in mouse model. Cell Mol Biol. (2012) 58(Suppl.):OL1646–53. 22455981

[13] DuttaAGuptaMLKalitaB. The combination of the active principles of Podophyllum hexandrum supports early recovery of the gastrointestinal system via activation of Nrf2-HO-1 signaling and the hematopoietic system, leading to effective whole-body survival in lethally irradiated mice. Free Radic Res. (2015) 49:317–30. 10.3109/10715762.2015.100432825564093

[14] SrivastavaNNShuklaSKYashavarddhanMHDeviMTripathiRPGuptaML. Modification of radiation-induced DNA double strand break repair pathways by chemicals extracted from *Podophyllum hexandrum*: an *in vitro* study in human blood leukocytes. Environ Mol Mutagen. (2014) 55:436–48. 10.1002/em.2185324500925

[15] DuttaSYashavarddhanMHSrivastavaNNRanjanRBajajSKalitaB. Countering effects of a combination of podophyllotoxin, podophyllotoxin beta-D-glucoside and rutin hydrate in minimizing radiation induced chromosomal damage, ROS and apoptosis in human blood lymphocytes. Food Chem Toxicol. (2016) 91:141–50. 10.1016/j.fct.2016.03.00726993954

[16] VermaSGuptaML. Radiation-induced hematopoietic myelosuppression and genotoxicity get significantly countered by active principles of *Podophyllum hexandrum*: a study in strain 'A' mice. Int J Radiat Biol. (2015) 91:757–70. 10.3109/09553002.2015.106257626073527

[17] GanieSAAminSHamidRHamidAMajeedRQurishiY. Podophyllum hexandrum aqueous extract as a potential free radical scavenger. Redox Rep. (2012) 17:54–62. 10.1179/1351000212Y.000000000422564348PMC6837480

[18] GuptaMLTyagiSFloraSJAgrawalaPKChoudharyPPuriSC. Protective efficacy of semi purified fraction of high altitude podophyllum hexandrum rhizomes in lethally irradiated Swiss albino mice. Cell Mol Biol. (2007) 53:29–41. 17543231

[19] SinghAYashavarddhanMHKalitaBRanjanRBajajSPrakashH. Podophyllotoxin and rutin modulates ionizing radiation-induced oxidative stress and apoptotic cell death in mice bone marrow and spleen. Front Immunol. (2017) 8:183. 10.3389/fimmu.2017.0018328289414PMC5326804

[20] VermaSKalitaBBajajSPrakashHSinghAKGuptaML. A combination of podophyllotoxin and rutin alleviates radiation-induced pneumonitis and fibrosis through modulation of lung inflammation in mice. Front Immunol. (2017) 8:658. 10.3389/fimmu.2017.0065828649248PMC5465247

[21] FujiwaraNKobayashiK. Macrophages in inflammation. Curr Drug Targets Inflamm Allergy (2005) 4:281–6. 10.2174/156801005402202416101534

[22] SicaAErreniMAllavenaPPortaC. Macrophage polarization in pathology. Cell Mol Life Sci. (2015) 72:4111–26. 10.1007/s00018-015-1995-y26210152PMC11113543

[23] DevittAMarshallLJ. The innate immune system and the clearance of apoptotic cells. J Leukoc Biol. (2011) 90:447–57. 10.1189/jlb.021109521562053

[24] NadellaVWangZJohnsonTSGriffinMDevittA. Transglutaminase 2 interacts with syndecan-4 and CD44 at the surface of human macrophages to promote removal of apoptotic cells. Biochim Biophys Acta (2015) 1853:201–12. 10.1016/j.bbamcr.2014.09.02025449226

[25] GordonS. The role of the macrophage in immune regulation. Res Immunol. (1998) 149:685–8. 10.1016/S0923-2494(99)80039-X9851524

[26] TabasIBornfeldtKE. Macrophage phenotype and function in different stages of atherosclerosis. Circ Res. (2016) 118:653–67. 10.1161/CIRCRESAHA.115.30625626892964PMC4762068

[27] MartinezFOGordonS. The M1 and M2 paradigm of macrophage activation: time for reassessment. F1000Prime Rep. (2014) 6:13. 10.12703/P6-1324669294PMC3944738

[28] GalliSJBorregaardNWynnTA. Phenotypic and functional plasticity of cells of innate immunity: macrophages, mast cells and neutrophils. Nat Immunol. (2011) 12:1035–44. 10.1038/ni.210922012443PMC3412172

[29] ItalianiPBoraschiD. From monocytes to M1/M2 macrophages: phenotypical vs. functional differentiation. Front Immunol. (2014) 5:514. 10.3389/fimmu.2014.0051425368618PMC4201108

[30] DasASinhaMDattaSAbasMChaffeeSSenCK. Monocyte and macrophage plasticity in tissue repair and regeneration. Am J Pathol. (2015) 185:2596–606. 10.1016/j.ajpath.2015.06.00126118749PMC4607753

[31] SicaAMantovaniA. Macrophage plasticity and polarization: *in vivo* veritas. J Clin Invest. (2012) 122:787–95. 10.1172/JCI5964322378047PMC3287223

[32] PrakashHAliABalaMGoelHC. Anti-inflammatory effects of *Podophyllum hexandrum* (RP-1) against lipopolysaccharides induced inflammation in mice. J Pharm Pharm Sci. (2005) 8:107–14. 15946604

[33] SchaueDKachikwuELMcBrideWH. Cytokines in radiobiological responses: a review. Radiat Res. (2012) 178:505–23. 10.1667/RR3031.123106210PMC3723384

[34] DiMaggio FMMinafraLForteGICammarataFPLioDMessaC Portrait of inflammatory response to ionizing radiation treatment. J Inflamm. (2015) 12:14 10.1186/s12950-015-0058-3PMC433676725705130

[35] GoelHCPrakashHAliABalaM. Podophyllum hexandrum modulates gamma radiation-induced immunosuppression in Balb/c mice: implications in radioprotection. Mol Cell Biochem. (2007) 295:93–103. 10.1007/s11010-006-9277-517029008

[36] GengozianNTaylorTJamesonHLeeETGoodRAEpsteinRB. Radiation-induced hemopoietic death in mice as a function of photon energy and dose rate. Radiat Res. (1986) 105:320–7. 10.2307/35766883961097

[37] WangNLiangHZenK. Molecular mechanisms that influence the macrophage m1-m2 polarization balance. Front Immunol. (2014) 5:614. 10.3389/fimmu.2014.0061425506346PMC4246889

